The article "Permanent Cardiac Sarcomere Changes in a Rabbit Model of Intrauterine Growth Restriction" was published in 2014. Journal: PLoS One.

# Permanent Cardiac Sarcomere Changes in a Rabbit Model of Intrauterine Growth Restriction

**DOI:** 10.1371/journal.pone.0113067

**Published:** 2014-11-17

**Authors:** Iratxe Torre, Anna González-Tendero, Patricia García-Cañadilla, Fátima Crispi, Francisco García-García, Bart Bijnens, Igor Iruretagoyena, Joaquin Dopazo, Ivan Amat-Roldán, Eduard Gratacós

**Affiliations:** 1 BCNatal – Barcelona Center for Maternal-Fetal and Neonatal Medicine (Hospital Clínic and Hospital Sant Joan de Deu), IDIBAPS, University of Barcelona, and Centre for Biomedical Research on Rare Diseases (CIBER-ER), Barcelona, Spain; 2 Physense, Departament de Tecnologies de la Informació i les Comunicacions (DTIC), Universitat Pompeu Fabra, Barcelona, Spain; 3 Bioinformatics Department, Centro de Investigación Principe Felipe (CIPF), Valencia, Spain; 4 Functional Genomics Node, INB, CIPF, Valencia, Spain; 5 Centro de Investigación Biomédica en Red de Enfermedades Raras (CIBERER), CIPF, Valencia, Spain; 6 ICREA, Universitat Pompeu Fabra, Barcelona, Spain; University of Southampton, United Kingdom

## Abstract

**Background:**

Intrauterine growth restriction (IUGR) induces fetal cardiac remodelling and dysfunction, which persists postnatally and may explain the link between low birth weight and increased cardiovascular mortality in adulthood. However, the cellular and molecular bases for these changes are still not well understood. We tested the hypothesis that IUGR is associated with structural and functional gene expression changes in the fetal sarcomere cytoarchitecture, which remain present in adulthood.

**Methods and Results:**

IUGR was induced in New Zealand pregnant rabbits by selective ligation of the utero-placental vessels. Fetal echocardiography demonstrated more globular hearts and signs of cardiac dysfunction in IUGR. Second harmonic generation microscopy (SHGM) showed shorter sarcomere length and shorter A-band and thick-thin filament interaction lengths, that were already present *in utero* and persisted at 70 postnatal days (adulthood). Sarcomeric M-band (GO: 0031430) functional term was over-represented in IUGR fetal hearts.

**Conclusion:**

The results suggest that IUGR induces cardiac dysfunction and permanent changes on the sarcomere.

## Introduction

Intrauterine growth restriction (IUGR) is a major cause of perinatal mortality and long term morbidity [1] affecting up to 7–10% of pregnancies. IUGR results in low birth weight, which has been epidemiologically associated with an increased risk of cardiovascular disease in adulthood [2]. This association is thought to be mediated through fetal cardiovascular programming. Fetuses with IUGR suffer from chronic oxygen and nutrients restriction [3], which triggers an adaptive hemodynamic cardiovascular adaptation [4], [5] associated with *in utero* volume and pressure overload [6]. Consequently, IUGR fetuses and newborns show signs of cardiovascular remodelling and dysfunction, including reduced annular peak velocities [7] and increased carotid intima-media thickness [8]. These fetal changes persist postnatally, as shown in human children [9] and in adult animal models [10], [11]. Although the effects of IUGR on cardiac organ remodelling have been characterized, the features of cardiac fetal programming at subcellular scale are poorly documented. Identifying cellular and molecular pathways involved in the fetal cardiac programming may provide a better understanding into the pathogenesis of the disease and could be an opportunity to design therapeutic interventions reducing the burden of cardiovascular disease from early life.

The article "Permanent Cardiac Sarcomere Changes in a Rabbit Model of Intrauterine Growth Restriction" was published in 2014. Journal: PLoS One.

The sarcomere is the basic functional unit of the cardiac contractile machinery. Changes in sarcomere structure and its key proteins have been observed in experimental models of cardiac dysfunction and failure [12]–[14]. In a previous study, we demonstrated that chronic pre-natal hypoxia induced permanent post-natal changes in the content and isoforms of sarcomeric proteins, including titin and myosin [10]. Interestingly, in another recent study in human hearts, we have demonstrated that severe IUGR fetuses present signs of cardiac dysfunction associated with changes in sarcomere length [15]. Sarcomere length is strongly related to sarcomere function and contraction force, and has been described to be consistently altered in a substantial number of conditions associated with cardiac failure [16]–[18].

In the current study, we aimed to evaluate the long term impact of IUGR on sarcomere structure in an experimental rabbit model of IUGR previously described by our group [19] that reproduces the main biometric and cardiovascular features of human IUGR. Hearts from IUGR fetuses as well as hearts from young adult rabbits were evaluated in order to assess the postnatal persistence of the changes on sarcomere architecture. Additionally, gene expression analysis of the fetal hearts combined with the functional interpretation of the global gene expression profile were assessed to gain further insight on changes in pathways and proteins regulating the sarcomere.

## Methods

### Experimental model of IUGR

New Zealand White rabbits were provided by a certified breeder and housed for 1 week before surgery in separate cages on a reversed 12/12 h light cycle. Dams were fed a diet of standard rabbit chow and water *ad libitum.* Animal handling and all procedures were carried out in accordance to applicable regulations and guidelines and with the approval of the Animal Experimental Ethics Committee of the University of Barcelona (permit number: 310/11–5999) and all efforts were made to minimize suffering.

The article "Permanent Cardiac Sarcomere Changes in a Rabbit Model of Intrauterine Growth Restriction" was published in 2014. Journal: PLoS One.

Ten New Zealand White pregnant rabbits were used to reproduce a previously described experimental model of IUGR [19], [20]. Briefly, at 25 days of gestation dams were intramuscularly administered ketamine 35 mg/kg and xylazine 5mg/kg for anesthesia induction. Tocolysis (progesterone 0,9 mg/kg intramuscularly) and antibiotic prophylaxis (Penicillin G 300.000 UI endovenous) were administered prior to surgery. Rabbits have two uterine horns, which were exteriorized after a midline laparatomy. Randomly, one uterine horn was denominated as the IUGR horn, while the other as the control horn. In all gestational sacs from the IUGR horn, a selective ligature of the 40–50% of the uteroplacental vessels of each gestational sac was performed. No ligature was performed in the control horn in order to subject control animals to the same anaesthetic and surgical procedures than the IUGR animals. The abdomen was then closed and animals received subcutaneous meloxicam 0.4 mg/kg/24 h for 48 h, as postoperative analgesia. Five days after surgery, the same anaesthetic procedure was applied to perform a caesarean section. At this moment, fetal echocardiography was performed. Subsequently, rabbit kits were obtained and randomly assigned to two age study groups: fetal (30 days of gestation) and young adult (70 days post-natal) group. Hearts from rabbits included in the fetal group were obtained through a thoracotomy after anesthesia. Hearts for gene expression study were immediately snap frozen and stored at −80°C until use. Hearts for multiphoton microscopy imaging were arrested in Ca^2+^-free buffer and fixed in 4% paraformaldehyde in phosphate buffer for 24 hours at 4°C. Fetuses included in the young adult group were breast-fed by a wet-nurse rabbit until the age of 25 days. At the age of 70 postnatal days, animals were anesthetized and hearts were excised and fixed in 4% paraformaldehyde in phosphate buffer.

### Fetal echocardiography

Echocardiography was performed in 10 paired control and IUGR rabbit fetuses at the time of the caesarean section by placing the probe directly on the uterine wall using a Vivid q (General Electric Healthcare, Horten, Norway) 4.5–11.5 MHz phased array probe. The angle of insonation was kept <30° in all measurements and a 70 Hz high pass filter was used to avoid slow flow noise. Ultrasound evaluation included: (1) Ductus venosus pulsatility index obtained in a midsagittal section or transverse section of the fetal abdomen positioning the Doppler gate at its isthmic portion; (2) Aortic isthmus pulsatility index obtained in a sagittal view of the fetal thorax with a clear view of the aortic arch placing the sample volume between the origin of the last vessel of aortic arch and the aortic joint of the ductus arteriosus; (3) Left and right sphericity indices calculated as base-to-apex length/basal ventricular diameter measured from 2-dimensional images in an apical 4-chamber view at end-diastole; (4) Left ventricular free wall thickness measured by M-mode in a transverse 4-chamber view; (5) Left ejection fraction estimated by M-mode from a transverse 4-chamber view according to Teicholz formula; (6) Longitudinal systolic (S') peak velocities at the mitral annulus measured by spectral tissue Doppler from an apical 4-chamber view.

The article "Permanent Cardiac Sarcomere Changes in a Rabbit Model of Intrauterine Growth Restriction" was published in 2014. Journal: PLoS One.

### Second Harmonic Generation Microscopy (SHGM)

Fixed fetal and young adult hearts were dehydrated and embedded in paraffin. Transversal 30 µm heart sections were cut in a microtome (Leica RM 2135) and mounted onto silane coated thin slides. After deparaffination with xylene and hydration with decreasing ethanol concentrations (100°/96°/70°), sections were covered with Mowiol 4–88 mounting medium (Sigma-Aldrich).

Detection of SHGM, from unlabelled cardiac tissue samples which were identified to contain mostly cardiomyocytes and no collagen, was performed with a Leica TCS-SP5 laser scanning spectral confocal multiphoton microscope (Leica Microsystems Heidelberg GmbH, Manheim, Germany) equipped with a Near Infrared laser (Mai Tai Broad Band 710–990 nm, 120 fempto second pulse), at the Advanced Optical Microscopy Unit from Scientific and Technological Centres from University of Barcelona. 7 control and 7 IUGR hearts from both the fetal and the young adult group were included in the analysis. For each heart, between 8 and 10 SHGM images, randomly chosen from the left ventricular mid-wall, were acquired. Each image included an average of 15 cardiac muscle fibers containing 200 sarcomeres approximately. The image resolution was 40 nm/pixel. Left ventricular cardiac fibers, which are mostly oriented in a single axis in optical sections of approximately 1.5 microns, were aligned at 45 degrees to maximize Signal to Noise Ratio (SNR) of SHGM. All tissue sections consisted of almost parallel fibres and were contained in a single plane by the sample preparation to avoid any bias in measurements. This certified that the statistical differences are related to group differences and contributions from other source of experimental error are marginal.

**Figure 1** shows the distinctive biperiodic pattern of sarcomeres, imaged by means of SHGM, and their characterization by two distances in unstained intact sarcomeres: resting sarcomere lengths (SL), measured as the distance between the two Z-discs delimiting each sarcomere; and intra-sarcomeric A-band lengths (ABL), defined as the distance between the two intra-sarcomeric segments of the A-band, divided by the M-band. Additionally, since SHGM arises from the thick-thin filament overlap in mature and developing sarcomeres [21], its length was calculated as the mean width of the A-band-related peak (namely in our study as thick-thin filament interaction length; TTIL). The three distinctive sarcomere distances (SL, ABL and TTIL) were measured automatically with a custom algorithm based on an optimal fitting of a parametric model of the autocorrelation function of the SHGM intensity profile in sarcomere fibers, as previously reported [22]. Briefly, the local orientation of the sarcomere fibers was estimated to perform automatically the following tracking of all the fibers within an image. After that, the SHGM intensity profile within each fiber was obtained and its autocorrelation function was computed. Finally, the autocorrelation function of the intensity profile was fitted with a parametric model to extract the average SL, ABL and TTIL of all the sarcomeres in the fiber. This calculation was performed for all the sarcomere fibers in the image. Additionally, a ratio between SL and ABL was calculated to further assess the quality of the acquired images and comparable physiological conditions between study groups. When this ratio was above 2.25, the sample was excluded from the analysis since the typical SHGM pattern of cardiac sarcomeres was lost.

The article "Permanent Cardiac Sarcomere Changes in a Rabbit Model of Intrauterine Growth Restriction" was published in 2014. Journal: PLoS One.

**Figure 1:** Schematic representation of the sarcomere cytoskeleton distances. **A**, an illustration of the sarcomere elementary parts; **B**, a sarcomere image by electron microscopy; **C**, a SHGM image of a myofibril; and **D**, a SHGM intensity profile along the myofibril showing the distances measured to characterize the sarcomere cytoskeleton: sarcomere length (SL), intra-sarcomeric A-band lengths (ABL) and thick-thin filament interaction length (TTIL).

### Gene expression microarray

The gene expression profile was analyzed in 6 paired control and IUGR rabbit fetal hearts at 30 days of gestation as previously described [23]. This study focused on the expression profile of the cardiomyocyte contractile machinery – the sarcomere. Total RNA was isolated from left ventricle (RNeasy Mini kit, Qiagen), labelled with Quick Amp One-color Labelling kit (Agilent) and fluorochrome Cy3 and hybridized with a Rabbit Microarray (Agilent Microarray Design ID 020908). The hybridization was quantified at 5 µm resolution (Axon 4000B scanner) and data extraction was performed using Genepix Pro 6.0. Data obtained from the microarray were pre-processed and subjected to bioinformatics analysis from two viewpoints. Firstly, a differential gene expression analysis in order to identify up- or down-regulated individual genes associated with IUGR, carried out using the *limma* [24] package from Bioconductor (http://www.bioconductor.org/). Differential gene expression of the samples in each group was assessed with the adjusted P value for every gene included in the microarray and with the fold change. Multiple testing adjustments of p-values were done according to Benjamini and Hochberg [25] methodology. All the pre-processing steps described can be carried out with the Babelomics software [26].

The article "Permanent Cardiac Sarcomere Changes in a Rabbit Model of Intrauterine Growth Restriction" was published in 2014. Journal: PLoS One.

Secondly, a gene set analysis was carried out for the Gene Ontology (GO) annotations using FatiScan [27] algorithm, implemented in the Babelomics suite [28], as previously described [23]. Briefly, FatiScan is able to detect up or down-regulated blocks of functionally related genes within the lists of genes originated in the microarray experiment, which are ordered by differential expression. The algorithm uses various criteria to look for modules of genes that are functionally related, such as GO terms. Within the whole list of genes, FatiScan evaluates the distribution of functional terms and extracts GO terms that are significantly under- and over-represented. GO terms are grouped in three classes: i) cellular components; ii) biological processes and iii) molecular functions. In order to compare the two groups of genes and extract a list of GO terms whose distribution among the groups is significantly different, FatiScan uses a Fisher's exact test for 2×2 contingency tables and a multiple test correction to finally obtain an adjusted p-value.

GO annotations for the genes in the microarray where taken from Blast2GO Functional Annotation Repository web page (http://bioinfo.cipf.es/b2gfar/) [29].The raw microarray data is deposited in the Gene Expression Omnibus database under accession number GSE37860.

### Statistical Analysis

Data were analyzed with the statistical package SPSS 15.0 (version 15.0; SPSS Inc, Chicago, IL). Data are expressed as mean ± standard deviation or median (Interquartile range (IQR)). Paired comparisons between the control and IUGR groups were done with t-test analysis. A classical parametric ANOVA test was carried out to compute significance between IUGR and control populations in experiments concerning SHGM analysis. Differences were considered significant with probability values of p<0.05. Statistical methods related to the gene expression analysis have been detailed in its previous corresponding section.

The article "Permanent Cardiac Sarcomere Changes in a Rabbit Model of Intrauterine Growth Restriction" was published in 2014. Journal: PLoS One.

## Results

### Fetal biometric and echocardiographic results

**Table 1** details the fetal biometric and echocardiographic data. While absolute fetal body and heart weights were significantly lower in IUGR, heart to body weight ratio was significantly increased in IUGR fetuses as compared to controls. Fetal echocardiography showed a more globular cardiac shape with lower right sphericity index but similar wall thickness in IUGR as compared to controls. Despite similar results in ejection fraction, mitral annular peak velocities (S') were significantly lower in IUGR as compared to controls. Additionally, ductus venosus and aortic isthmus pulsatility indices were significantly increased in IUGR fetuses.

**Table 1:** Fetal biometric and echocardiographic results in IUGR and control fetuses.

	Control	IUGR	P-value
N	10	10	
**Fetal Biometry**			
Fetal weight (g)	48.97 (12.46)	29.94 (7.72)	0.000 *
Heart weight (g)	0.37 (0.10)	0.29 (0.09)	0.006 *
Heart weight/Fetal weight)*100	0.79 (0.11)	1.10 (0.31)	0.009 *
**Fetal hemodynamics**			
Ductus venosus pulsatility index	0.75 (0.25)	1.33 (0.75)	0.008 *
Aortic isthmus pulsatility index	3.05 (0.45)	3.85 (1.16)	0.009 *
**Cardiac morphometry**			
Left sphericity index	1.54 (0.34)	1.51 (0.26)	0.073
Right sphericity index	1.56 (0.24)	1.32 (0.23)	0.004 *
Left ventricle wall thickness (mm)	1.45 (0.37)	1.41 (0.31)	0.978
**Systolic function**			
Left ejection fraction (%)	89.1 (8.2)	82 (24.6)	0.39
Mitral annular systolic peak velocity (cm/s)	1.91 (0.27)	1.59 (0.33)	0.046 *

All values are median (interquartile range). P-value was calculated by t-test. *g:* grams; *mm:* millimeters; *cm/s*: centimetres/second. * P-value <0.05.

### Fetal sarcomere morphometry

Seven paired control and IUGR rabbits were quantified demonstrating a readily detectable SHGM signal from unstained left ventricular sarcomeres. A representative image is displayed in **Figure 2A** and a magnification of it is shown in **Figure 1**.

**Figure 2:** Ultrastructural sarcomere changes in fetal hearts from IUGR and controls. **A,** A representative SHGM image from unstained fetal rabbit left ventricle. The sarcomeres are clearly delimited by thick black lines (Z-discs) and the SHGM signal originates from the thick myosin filaments (in green). In the central region of the myosin filaments appears a thinner black line, identified as the M-band. Scale bar = 20 µm. **B** and **C,** show average distances between two consecutive Z-discs (SL) and intrasarcomeric A-bands (ABL), respectively. **D,** shows thick-thin filament interaction length (TTIL), as the mean width of the A-band-related peaks. Data are expressed as mean ± SD.

The article "Permanent Cardiac Sarcomere Changes in a Rabbit Model of Intrauterine Growth Restriction" was published in 2014. Journal: PLoS One.

As compared with controls, IUGR fetuses showed shorter sarcomere length (controls: 1.658 µm ±0.094 vs. IUGR 1.531 µm ±0.114, p = 0.042) (**Figure 2B**). Intra-sarcomeric A-band length was also found to be decreased by IUGR (controls 0.772 µm ±0.044 vs. IUGR 0.705 µm ±0.060, p = 0.035) (**Figure 2C**). Additionally, thick-thin filament interaction length was shorter in IUGR (controls 0.104 µm ±0.006 vs. IUGR 0.096 µm ±0.007, p = 0.048) (**Figure 2D**). The ratio between sarcomere length and intrasarcomeric A-band length was similar in the study groups (controls 2.15±0.02 vs. IUGR 2.17±0.03).

### Post-natal persistence of cardiac sarcomeric changes

Unstained young adult rabbit sarcomeres from left ventricular samples, in seven paired control and IUGR rabbits (70 postnatal days), produced a readily detectable SHGM signal (**Figure 3A**) with a pattern similar to the one observed in fetal sarcomeres, with similar ratios between sarcomere length and intrasarcomeric A-band length (controls 2.11±0.02 vs. IUGR 2.11±0.01). A significant decrease in sarcomere length (controls 1.720 µm ±0.068 vs. IUGR 1.626 µm ±0.084, p = 0.04) and intrasarcomeric A-band length (controls 0.817 µm ±0.036 vs. IUGR 0.772 µm ±0.041, p = 0.049) were observed in IUGR as compared to controls (**Figure 3B, C**). Additionally, sarcomeric thick-thin filament interaction length was shorter in IUGR (controls 0.103 µm ±0.005 vs. IUGR 0.097 µm ±0.005, p = 0.045) as compared to controls (**Figure 3D**).

**Figure 3:** Ultrastructural sarcomere changes in adult hearts from IUGR and controls. **A,** Representative SHGM image from unstained adult rabbit left ventricle. Scale bar  = 20 µm. **B** and **C,** show average distances between two consecutive Z discs (SL) and two intrasarcomeric A bands (ABL), respectively. **D,** shows the length of thick-thin filament interaction length (TTIL). Data are expressed as mean ± SD.

### Bioinformatic analysis of gene expression microarray data

#### Differential gene expression

All experiments showed a good level of labelling and hybridization onto the Agilent microarray. Differential gene expression (when analysing for a fold change higher than 0.5 and an adjusted p-value lower than 0.05– data not shown) was similar in both experimental conditions for all the cardiomyocyte sarcomere components included in the microarray.

#### Gene set analysis: functional interpretation of microarray data

A statistically significant enrichment in the group of genes composing the sarcomeric *M-band* (GO: 0031430) functional class (P raw <0.001; P adj  = 0.069) was observed in fetal IUGR hearts. The GO cellular component M-band is represented in **Figure 4** as an acyclic graph. *M band* annotation was found in 1.6% of the most up-regulated genes in IUGR. On the other hand, only 0.69% of the most down-regulated genes in IUGR contained the annotation (p value <0.001; adjusted p-value <0.1). **Table 2** shows the most relevant genes that define the *M band* (GO: 0031430). The remaining sarcomeric functional terms identified by the gene set analysis were not found to be significantly modified due to IUGR.

The article "Permanent Cardiac Sarcomere Changes in a Rabbit Model of Intrauterine Growth Restriction" was published in 2014. Journal: PLoS One.

**Figure 4:** Gene ontology analysis. Acyclic graph showing the M-line cellular component significantly over-represented (in red) in IUGR compared to healthy control hearts. In the GO hierarchy, biological knowledge can be represented as a tree where functional terms near the root of the tree make reference to more general concepts while deeper functional terms near the leaves of the tree make reference to more specific concepts. If a gene is annotated to a given level, then is automatically considered to be annotated at all the upper levels up to the root.

**Table 2:** Results from most relevant sequences included in M-band functional class identified by FatiScan gene set analysis (M-band (GO: 0031430) block of genes).

Name	ID	Fold change
OBSCN (Obscurin)	ENSOCUT00000011554	0.266
OBSL (Obscurin-like protein 1)	ENSOCUT00000011142	0.171
Titin	ENSOCUT00000016899	0.265
Myopalladin	ENSOCUT00000009940	0.405
Myomesin-2	ENSOCUT00000013143	0.265

A fold change value above 0 indicates up-regulation in IUGR vs. controls.

## Discussion

The present study shows an association between IUGR and fetal and postnatal permanent sarcomeric structural changes together with altered fetal cardiac function and sarcomere related gene expression changes. Since sarcomere length has been shown to have an important influence on cardiac contractility [30], the observed decrease in its length might be an important determinant of the currently described changes on cardiac shape and function. These findings provide important clinical and research suggestions that open future research to further characterize the molecular basis of cardiac dysfunction and remodelling observed in IUGR individuals.

The experimental approach used in this study chronically reduces the blood supply to the fetuses by performing a selective ligature of the uteroplacental vessels in pregnant rabbits [19], and has been shown to reproduce the main biometric and fetal hemodynamic features observed in human growth restriction [20]. Signs of fetal hypoxia are demonstrated by an increased pulsatility in the aortic isthmus flow as a reflection of the shift of blood towards the brain circulation in response to hypoxia, which is produced by a combination of brain vasodilation and systemic hypertension [31]. Additionally, the echocardiographic evaluation confirmed that IUGR results in more globular hearts, together with signs of systolic longitudinal dysfunction, which is similar to those changes observed in human fetuses and children [7], [9], [32].

The article "Permanent Cardiac Sarcomere Changes in a Rabbit Model of Intrauterine Growth Restriction" was published in 2014. Journal: PLoS One.

Sarcomere length is important in myofilament force generation by different mechanisms since it has an effect on actin-myosin cross-bridge recruitment [33]. In this regard, sarcomere length is associated with the degree of thick-thin filament overlap, which affects the probability of actin-myosin cross-bridge formation and thus the capacity to generate force [34]. Shorter sarcomeres have been found in animal models of a variety of cardiac diseases, including ischemic contracture [16], diastolic dysfunction [17], dilated cardiomyopathy and heart failure [18]. Additionally, in a recent paper using human biopsies, passive force-length analysis suggested a shorter sarcomere length in pressure-overloaded myocardium compared to volume overload and control donors [35]. We recently described changes on the cardiomyocyte intracellular organization in the same experimental animal model of IUGR [23] that resemble to changes induced by pressure overload [36]. The permanent changes in sarcomere structure, as observed here in IUGR, could be as well a response to the known sustained increase in fetal blood pressure that occurs in IUGR. Supporting this notion, recent findings suggest that isolated neonatal cardiomyocytes undergo structural modifications within their myofibrils in response to changes in environmental stiffness, resulting in differences in resting sarcomere length [37]. Additionally, the observed changes in sarcomere length are consistent with previous research where we showed that chronic prenatal hypoxia led to a shift in the expression of titin isoform N2BA (larger and more compliant isoform) towards isoform N2B (smaller and stiffer isoform) [10]. This protein extends from the center of the sarcomere to the *Z* line, thus acting as a developmental template for sarcomere assembly [38]. Titin is thought to be a major determinant of the sarcomere length [39], [17].

We recently published a work in which post-mortem cardiac samples from human fetuses that suffered severe IUGR were studied using the same SHGM methodology in order to assess changes in sarcomere morphometry [15]. Interestingly, results were strongly consistent with the ones described herein in the animal model: shorter sarcomere length in IUGR. This consistency strengthens the hypothesis that changes in sarcomere length could help to explain subclinical cardiac dysfunction previously described in human fetuses and children [9], and observed in IUGR rabbits in this study. The shorter sarcomere and thick-thin filament interaction length might indicate a decrease in the number of binding events for cross-bridges between actin and myosin. Since cardiac muscle energy consumption depends on the number of recruited cross-bridges [40] shorter sarcomere length and thick-thin filament interaction length could be interpreted as an adaptive mechanism to cope with the oxygen and/or glucose restriction in IUGR. Importantly, in this study we show evidence of the postnatal persistence of the changes on sarcomere morphometry, which can not be assessed in humans. This observation might be relevant to explain the increased risk of cardiovascular disease and mortality in adult life related to IUGR as well as to understand the fetal cardiac programming.

The article "Permanent Cardiac Sarcomere Changes in a Rabbit Model of Intrauterine Growth Restriction" was published in 2014. Journal: PLoS One.

Advanced bioinformatics analytic approaches were used in this study to complement the observations of SHGM and provide further evidence of the existence of functional gene expression differences encompassing structural changes. Fetal gene set analysis included a family of different tests designed to detect modules of functionally-related genes [41], [42]. Among them, we used FatiScan [27], integrated in Babelomics [26], which has been employed to successfully detect coordinated variations in blocks of genes [43]. The results demonstrated functional differences in a basic structure for the sarcomeric cytoskeleton, the M-band, which plays an important organizational role during myofibrillogenesis by performing the regular packing of the nascent thick (myosin) filaments [44]. This finding is in line with previous observations suggesting that specific structural alterations at the M-band might be part of a general adaptation of the sarcomeric cytoskeleton to unfavorable working conditions in early stages of dilated cardiomyopathy, correlating with an impaired ventricular function [45]. Moreover, they suggest an underlying basis for the abnormal sarcomere cytoarchitecture observed in IUGR. Genes included in the M-band functional class involve a variety of associated molecules to this structure with key roles in sarcomere assembly and function, including titin, obscurin and myomesin. Interference with the physiological function of these proteins is of pathogenic relevance for human cardiomyopathies [46]. The findings warrant further investigation to clarify the individual role of sarcomere proteins in the generation of permanent structural changes of the contractile machinery under IUGR.

Several study limitations and technical considerations merit discussion. We used SHGM to measure sarcomere length. The technique has been validated to accurately visualize the SHGM signal produced by cardiac myosin thick filaments in unstained sarcomeres from different species with an accuracy of 20 nm [21], [22], [47]. SHGM offers comparable results to those provided by electron microscopy with the additional advantage of imaging larger tissue areas [22]. Sarcomere length values in this study were consistent with measurements using electron and light microscopy in fixed rabbit cardiomyocytes, and showed increasing values with cardiac maturation [48], [49]. Although the intrasarcomeric A-band length from the second harmonic generation signal changes little depending upon sarcomere contraction [21], we acknowledge the hearts not being arrested with potassium and fixed at a known transmural pressure as a potential limitation of this study. The bioinformatics analysis of gene expression data used herein has been shown to be useful for studying diseases like IUGR in which subtle differences are expected. This study illustrates the existence of sarcomere changes, but it provides a limited view of the mechanistic or molecular pathways underlying such changes. We acknowledge that with the present study is difficult to address the actual biological relevance of the gene expression and bioinformatics analysis and future studies are required to gain further insight on the relevance and to elucidate pathways that might be responsible for the observed changes. Additionally, results provided by bioinformatics gene set analysis strongly depend on the capabilities of bioinformatics tools and gene annotations, which are constantly evolving. Thus, gene pathways that are not well described yet might remain undetectable with current tools

In conclusion, this study provides new clues towards understanding the cellular and molecular mechanisms underlying cardiac remodelling through fetal programming and persisting in adulthood. Together, the findings presented here support that IUGR induces permanent changes in cardiac sarcomere morphometry, associated with functional changes in proteins involved in sarcomere function and assembly. These changes might help to explain the stiffer and less deforming hearts of fetuses and adults suffering from IUGR, and open new lines of research aiming at characterizing and interfering with the mechanisms of adaptation leading to cardiovascular remodelling in IUGR.
